The article "Decreased expression of the long noncoding RNA LINC00261 indicate poor prognosis in gastric cancer and suppress gastric cancer metastasis by affecting the epithelial–mesenchymal transition" was retracted in 2018. Reasons: duplicated images; unreliable data.

# Decreased expression of the long noncoding RNA LINC00261 indicate poor prognosis in gastric cancer and suppress gastric cancer metastasis by affecting the epithelial–mesenchymal transition

**DOI:** 10.1186/s13045-016-0288-8

**Published:** 2016-07-21

**Authors:** Yu Fan, Yan-fen Wang, Hua-fang Su, Na Fang, Chen Zou, Wen-feng Li, Zheng-hua Fei

**Affiliations:** Cancer Institute, The Affiliated People’s Hospital of Jiangsu University, Zhenjiang, Jiangsu 212002 People’s Republic of China; Department of Pathology, the First People’s Hospital of Yangzhou/The Second Clinical Medical College, Yangzhou University, Yangzhou, Jiangsu 225000 People’s Republic of China; Radiotherapy and Chemotherapy Department, The 1st Affiliated Hospital of Wenzhou Medical University, No.2 Fuxue Lane, 325000 Wenzhou, China

**Keywords:** LINC00261, Metastasis, Prognosis, Gastric cancer

## Abstract

**Background:**

Recent evidence indicates that long noncoding RNAs (lncRNAs) play pivotal roles in the regulation of cellular processes and are found to be dysregulated in a variety of cancers. LINC00261 is an lncRNA that is aberrantly expressed in gastric cancer (GC). The clinical role of LINC00261 in GC and molecular mechanisms remains to be found.

**Methods:**

Real-time polymerase chain reaction (PCR) was used to examine LINC00261 expression in GC cell lines/tissues compared with normal epithelial cells/adjacent non-tumorous tissues. Gain and loss of function approaches were used to investigate the biological role of LINC00261 in GC cells. The effects of LINC00261 on cell viability were evaluated by MTT and colony formation assays. Wound healing assay, cell migration and invasion assays, and nude mice were used to examine the effects of LINC00261 on tumor cell metastasis in vitro and in vivo. Protein levels of LINC00261 targets were determined by western blot and immunohistochemistry.

**Results:**

LINC00261 was downregulated in GC cell lines and cancerous tissues, as compared with normal gastric epithelial cells and adjacent noncancerous tissue samples. Low LINC00261 expression was correlated with deeper tumor invasion (*P* < 0.001), higher tumor stage (*P* = 0.013), and lymphatic metastasis (*P* = 0.006). Univariate and multivariate analyses indicated that low LINC00261 expression predicted poor prognosis. Ectopic expression of LINC00261 impaired cell migration and invasion, leading to the inhibition of metastasis in vitro and in vivo. Knockdown of LINC00261 expression promoted cell migration and invasion in vitro. Overexpression of LINC00261 was found to play a key role in epithelial–mesenchymal transition (EMT) through the regulation of E-cadherin, N-cadherin, and Vimentin expression.

The article "Decreased expression of the long noncoding RNA LINC00261 indicate poor prognosis in gastric cancer and suppress gastric cancer metastasis by affecting the epithelial–mesenchymal transition" was retracted in 2018. Reasons: duplicated images; unreliable data.

**Conclusions:**

Low expression of the lncRNA LINC00261 occurs in GC and is associated with poor prognosis. LINC00261 suppresses GC metastasis by regulating EMT. Thus, LINC00261 plays an important role in the progression and metastasis of GC.

**Electronic supplementary material:**

The online version of this article (doi:10.1186/s13045-016-0288-8) contains supplementary material, which is available to authorized users.

## Background

Gastric cancer (GC) represents the fourth most common malignancy in the world and second leading cause of cancer-related deaths worldwide, with particularly high frequencies in East Asia [1]. Although GC is curable if detected early, most patients are diagnosed in the advanced stage and have poor prognosis [2]. Tumor invasion and metastasis are the main causes accounting for the poor prognosis [3]. The clinical stage, based on the TNM classification system, at the time of diagnosis is currently the most important prognostic factor, and the molecular mechanism involved in the progression and metastasis of GC remains unknown [4]. Thus, novel prognostic factors that are associated with GC progression and metastasis would be of great clinical relevance.

Apart from about 2 % protein-coding genes, more than 90 % of the genome is transcribed as noncoding RNAs (ncRNAs), indicating that ncRNAs could play significant regulatory roles in complex organisms [5, 6]. One subcategory of these transcripts, called long noncoding RNAs (lncRNAs), comprises ncRNAs that are more than 200 nucleotides in length. Accumulating evidence demonstrates that lncRNAs play roles in a variety of biological processes, including chromatin remodeling, cell differentiation, and immune responses [7–9]. In addition, recent reports have showed that some lncRNAs exhibit distinct gene expression patterns and play significant roles during cellular development in various types of carcinomas [10–12]. However, the overall pathophysiological contributions of lncRNAs to gastric carcinoma remain largely obscure. Functional lncRNAs can be used for cancer diagnosis and prognosis and serve as potential therapeutic targets; thus, lncRNAs can be considered as a new diagnostic and therapeutic gold mine in cancer [13]. The lncRNA profiling study revealed that lncRNA LINC00261, an lncRNA mapped to 20p11.21, was found to be downregulated in GC tissues compared to normal tissue samples [14]. However, the role of LINC00261 in GC progression remains unknown.

In this study, we found that LINC00261 expression was reduced in GC tissues and cell lines. Low expression of LINC00261 was associated with clinicopathological characteristics and poor prognosis in GC patients. Ectopic expression of LINC00261 in gastric cells significantly inhibited cell migration and invasion. Conversely, depletion of LINC00261 promoted these activities. Moreover, we also showed that alteration of LINC00261 expression can influence E-cadherin, N-cadherin, Fibronectin1 (FN1), and Vimentin protein levels, which indicated that LINC00261 affected GC cell invasion and metastasis partly via epithelial–mesenchymal transition (EMT). These studies advance our understanding of the role of lncRNAs, such as LINC00261 as a regulator of pathogenesis of GC, and facilitate the development of lncRNA-directed diagnostics and therapeutics.

The article "Decreased expression of the long noncoding RNA LINC00261 indicate poor prognosis in gastric cancer and suppress gastric cancer metastasis by affecting the epithelial–mesenchymal transition" was retracted in 2018. Reasons: duplicated images; unreliable data.

## Results

### LINC00261 expression and clinicopathological factors in GC

A human lncRNA microarray dataset (GSE13911) (38 paired cancer and noncancer tissues) was obtained to analyze differentially expressed lncRNAs between GC and paired non-tumor tissues. Twenty lncRNAs had an obvious fold change in GC tissues when compared with corresponding non-tumor tissues as supplied in Table 1. LINC00261 expression levels were the most downregulated in this database (Fig. 1a), which is consistent with a previous report [14]. To ensure that conclusions derived from these results are reliable, we have compared the LINC00261 expression between paired GC and normal tissues (*n* = 138) and tested for statistical significance by Student’s paired *t* test. Analysis of tumor/non-tumor adjacent tissue (T/N) ratios for LINC00261 expression of 138 patients revealed that LINC00261 expression was decreased in approximately 80 % GC patient tissues (*P* < 0.001, Fig. 1b). Reverse transcription (RT)-qPCR assays were further developed to quantify LINC00261 in GC cell lines, including MGC803, BGC823, MKN28, MKN45, and SGC7901, and in the normal gastric epithelium cell line GES1. Significantly lower expression of LINC00261 was found in MKN28 (*P* = 0.008), MKN45 (*P* = 0.038), BGC823 (*P* = 0.003), SGC7901 (*P* = 0.022), and MGC803 (*P* = 0.045) than in GES-1 (Fig. 1c).

**Table 1:** Twenty candidate lncRNAs expressed with more than twofold changes compared with corresponding non-tumor tissues

Fold change	*P* value	FDR value	Gene name
5.3	<0.001	<0.001	*UCA1*
4.6	<0.001	<0.001	*H19*
4.8	<0.001	0.003269372	*HOXA11-AS*
4.0	<0.001	<0.001	*LOC100131046*
3.6	0.006	0.02	*BCAR4*
3.2	<0.001	<0.001	*LINC00152*
2.8	0.0055	0.019	*ANKRD30BP2*
2.6	<0.001	<0.001	*KRT16P2*
2.5	<0.001	<0.001	*HMGB3P1*
2.3	<0.001	<0.001	*SNHG10*
2.1	<0.001	<0.001	*SNHG5*
2.2	<0.001	<0.001	*HOTAIR*
2.2	<0.001	<0.001	*SPRR2C*
2.0	<0.001	<0.001	*MAFG-AS1*
0.50	<0.001	<0.001	*RP11-834C11.4*
0.42	<0.001	<0.001	*RP11-363E7.4*
0.35	<0.001	<0.001	*RP11-734 K23.9*
0.31	<0.001	<0.001	*RP11-160 N1.10*
0.23	<0.001	<0.001	*LINC00982*
0.18	<0.001	<0.001	*LINC00261*

The article "Decreased expression of the long noncoding RNA LINC00261 indicate poor prognosis in gastric cancer and suppress gastric cancer metastasis by affecting the epithelial–mesenchymal transition" was retracted in 2018. Reasons: duplicated images; unreliable data.

**Fig. 1:** Decreased expression of LINC00261 in gastric cancer tissues and cell lines. **a** LINC00261 expression is analyzed based on GSE13911 database. **b** Real-time PCR analysis of LINC00261 expression in normal gastric epithelial cell line (GES-1) and gastric cancer cells. Experiments were performed in triplicate. *Bars*: SD; *P < 0.05, **P < 0.01. **c** Examined LINC00261 expression by qRT-PCR in 138 paired human gastric cancer tissues and adjacent noncancerous tissues (paired *t* test, *P* < 0.001). Data are represented as log_2_-fold changes (cancer/normal), with “<−1” indicating underexpression and “>1” indicating overexpression. The patients were divided into a low LINC00261 expression group (69) and a high LINC00261 expression group (69), according to the median value of relative LINC00261 expression (3.8-fold, noncancerous/tumors). **d**, **e** ROC curves were conducted for prediction of gastric cancer tissues based on GSE13911 database and using qPCR-based LINC00261 expression level. The AUC was 0.921 (**d**) and 0.812 (**e**)

We plotted a receiver operating characteristic (ROC) curve with the non-tumorous tissues adjacent to the tumor tissues as a control based on the GSE13911 and our collected tissues. The cutoff value for predicting GC tissues from normal tissues was 5.22 (normalized intensity value) and 9.02 (*Δ* Ct value). The area under the ROC curve (AUC) was 0.921 (95 % confidence interval (CI) = 0.836–0.970, *P* < 0.001) and 0.812 (95 % CI = 0.743–0.869, *P* < 0.001) (Fig. 1d, e). The sensitivity and specificity were 0.97 and 0.87 and 0.76 and 0.75, respectively. To assess the correlation of LINC00261 expression with clinicopathological data, the expression levels of LINC00261 in tumor tissues were categorized as low or high in relation to the median value of relative LINC00261 expression (3.8-fold, noncancerous/tumors). Clinicopathological factors were analyzed in the high and low LINC00261 expression groups. As shown in Table 2, the low LINC00261 expression group (*n* = 69) showed greater invasion depth (*P* < 0.001), higher tumor stage (*P* = 0.013), and more frequent lymphatic metastasis (*P* = 0.006) than the high LINC00261 expression group (*n* = 69). However, there was no significant correlation between LINC00261 expression and other clinicopathological features such as age, sex, tumor location, tumor size, histological grade, and distant metastasis (*P* > 0.05). The clinical data of all patients is shown in Additional file 1: Table S2.

**Table 2:** Correlation between LINC00261 expression and clinicopathological characteristics of gastric cancer

Clinical parameter	LINC00261		Chi-squared test *P* value
	High-expression cases (*n* = 69)	Low-expression cases (*n* = 69)	
Age (years)			0.496
<50	33	37	
>50	36	32	
Gender			0.385
Male	39	44	
Female	30	25	
Location			0.561
Distal	29	30	
Middle	22	26	
Proximal	18	13	
Size			0.173
>5 cm	32	40	
<5 cm	37	29	
Histologic differentiation			0.206
Well	29	18	
Moderately	29	37	
Poorly	7	11	
Undifferentiated	4	3	
Invasion depth			<0.001*
T1	29	5	
T2	21	12	
T3	11	30	
T4	8	22	
TNM stages			0.013*
I	18	8	
II	26	19	
III	17	33	
IV	8	9	
Lymphatic metastasis			0.006*
Yes	41	25	
No	28	44	
Regional lymph nodes			<0.001*
PN0	42	25	
PN1	12	5	
PN2	9	22	
PN3	6	17	
Distant metastasis			0.796
Yes	8	9	
No	61	60	

*P < 0.05

The article "Decreased expression of the long noncoding RNA LINC00261 indicate poor prognosis in gastric cancer and suppress gastric cancer metastasis by affecting the epithelial–mesenchymal transition" was retracted in 2018. Reasons: duplicated images; unreliable data.

### LINC00261 is a bona fide ncRNA in GC

We first identified the full poly (A)-positive sequence of LINC00261 through rapid amplification of cDNA ends (RACE) and performed polymerase chain reaction (PCR) analysis to confirm the gene size of LINC00261. The RACE results identified two isoforms of LINC00261 (Additional file 2: Table S3). In addition, txCdsPredict, created by UCSC, was used to calculate its protein-coding potential, and a score was assigned based on its coding potential; we considered the transcript as ncRNA when the score was less than 800 [15]. The txCdsPredict score for LINC00261 was 245, indicating that LINC00261 has no protein-coding potential. We verified that LINC00261 was indeed an ncRNA through analysis of the sequences by ORF Finder from the National Center for Biotechnology Information and Coding Potential Calculator (CPC) [16]. ORF Finder failed to predict a protein of more than 205 amino acids (Fig. 2a), and the CPC score is −1.21477 (Fig. 2b). Moreover, LINC00261 does not contain a valid Kozak sequence, which further supports that LINC00261 has no protein-coding potential.

**Fig. 2:** LINC00261 is a long noncoding RNA. **a** Lack of open reading frame in the 4924-bp LINC00261 was verified by ORF Finder. **b** Coding Potential Calculator (CPC) showed that the CPC score of LINC00261is −1.21477, indicating LINC00261 has no coding protein potential

### Low LINC00261 expression is associated with poor prognosis in patients with GC

Kaplan–Meier analysis and log-rank test were used to evaluate the effects of LINC00261 expression and clinicopathological characteristics on disease-free survival (DFS). The results showed that patients in the low LINC00261 expression group had a higher recurrence rate (median DFS 19 months) than those in the high LINC00261 expression group (median DFS 35 months; *P* = 0.004; Fig. 3a). The 3-year DFS was 32.8 % in the low LINC00261 expression group, while 45.3 % in the high LINC00261 expression group. Moreover, the expression of LINC00261 was strongly correlated with DFS in the advanced clinical stages (stages III and IV; Fig. 3d, e). However, in patients in clinical stages I and II, no significant differences in DFS was found between those with low and high LINC00261 expression (Fig. 3b, c). Univariate analyses of clinical variables considered as potential predictors of survival are shown in Table 3. Further analysis in a multivariate Cox proportional hazards model showed that LINC00261 expression, together with TNM stage, was strongly associated with DFS. LINC00261 expression was an independent prognostic indicator of DFS (hazard ratio (HR) = 0.551; 95 % (CI), 0.323–0.940; *P* = 0.029) in patients with GC (Table 3).

The article "Decreased expression of the long noncoding RNA LINC00261 indicate poor prognosis in gastric cancer and suppress gastric cancer metastasis by affecting the epithelial–mesenchymal transition" was retracted in 2018. Reasons: duplicated images; unreliable data.

**Fig. 3:** The prognostic significance of LINC00261 in gastric cancer patients. **a** Kaplan–Meier analysis of disease-free survival (DFS) based on LINC00261 expression in all 138 patients. **b**–**e** Kaplan–Meier analysis of DFS based on LINC00261 expression in gastric cancer patients in stages I (**b**), II (**c**), III (**d**), and IV (**e**)

**Table 3:** Univariate and multivariate Cox regression analyses LINC00261 for DFS of patients in the study cohort (*n* = 138)

Variables	DFS		
	HR	95 % CI	*P* value
Univariate analysis			
Age (<50 vs. >50 years)	0.874	0.537–1.424	0.589
Gender (male vs. female)	0.802	0.484–1.329	0.392
Location (distal vs. middle + proximal)	0.793	0.487–1.292	0.351
Tumor size (>5 vs. <5 cm)	1.336	1.041–1.714	0.023*
Histologic differentiation (well + moderately vs. poorly + undifferentiated)	1.626	0.966–2.738	0.068
Invasion depth (T1 + T2 vs. T3 + T4)	1.174	0.721–1.911	0.518
TNM stage (III + IV vs. I + II)	2.620	1.561–4.395	<0.001*
Lymphatic metastasis (no vs. yes)	0.749	0.583–0.963	0.024*
Regional lymph nodes (PN2 + PN3 vs. PN0 + PN1)	1.818	1.111–2.972	0.017*
Distant metastasis (no vs. yes)	0.654	0.482–0.888	0.007*
Expression of LINC00261 (high vs. low)	0.494	0.300–0.812	0.005*
Multivariate analysis			
TNM stage (III + IV vs. I + II)	1.805	1.090–2.990	0.022*
Lymphatic metastasis (no vs. yes)	0.887	0.665–1.246	0.125
Regional lymph nodes (PN2 + PN3 vs. PN0 + PN1)	1.117	0.592–2.111	0.732
Tumor size (>5 vs. <5 cm)	1.086	0.835–1.433	0.510
Distant metastasis (no vs. yes)	0.584	0.294–1.162	0.126
Expression of LINC00261 (high vs. low)	0.551	0.323–0.940	0.029*

*P < 0.05

### LINC00261 exhibits an insignificant effect on GC cell proliferation, but represses GC cell migration and invasion in vitro

To gain further insight into the biologic pathways involved in GC pathogenesis stratified by the median of LINC00261 expression level, Gene Set Enrichment Analysis (GSEA) analysis was performed in GSE13911 datasets. Enrichment plots of GSEA showed that the gene signatures of cell adhesion were more correlated with patients with LINC00261 lower expression versus patients with LINC00261 higher expression in the dataset (Fig. 4a). The top-scoring genes recurring in the pathway included key cancer genes, such as E-cadherin, N-cadherin, CD44, matrix metalloproteinase (MMP)-2, MMP-9, and FN1 (Additional file 3: Table S4). Correlation analysis based on GSE13911 datasets showed that LINC00261 expression was positively correlated with E-cadherin and negatively related to N-cadherin and FN1 (Fig. 4b, c, d). Further real-time PCR data confirmed that alteration of LINC00261 expression dramatically affected the key gene signatures which are involved in tumor metastasis (Fig. 4e, f), suggesting that LINC00261 may be a key regulator in GC progression.

The article "Decreased expression of the long noncoding RNA LINC00261 indicate poor prognosis in gastric cancer and suppress gastric cancer metastasis by affecting the epithelial–mesenchymal transition" was retracted in 2018. Reasons: duplicated images; unreliable data.

**Fig. 4:** GSEA in LINC00261 higher/lower expression gastric cancer patients and the correlation between of LINC00261 and its target genes. **a** GSEA comparing LINC00261 lower expression group (*red*) against LINC00261 higher expression group (*blue*) of patients with gastric cancer in the GSE13911 dataset, illustrating distinct pathways and biologic processes between both subgroups. Enrichment plots are shown for a set of activated genes related to cell adhesion in GSE13911 patients’ dataset. The enrichment score (ES, *green line*) means the degree to which the gene set is overrepresented at the top or bottom of the ranked list of genes. *Black bars* indicate the position of genes belonging to the gene set in the ranked list of genes included in the analysis. A positive value indicates more correlation with “LINC00261 lower expression” patients and a negative value indicates more correlation with “LINC00261 higher expression” patients. **b**–**d** The Pearson correlation analysis of LINC00261 expression with target gene based on GSE13911 patients’ database. LINC00261 is negative related to FN1 (**b**) and N-cadherin (**d**), while positive correlated with E-cadherin (**c**). **e**, **f** qPCR analysis of LINC00261 expression levels following the treatment of BGC823 cells with empty vector and pcDNA3.1-LINC00261 (**e**), and the treatment of MGC803 cells with scrambled siRNA and si-LINC00261 (**f**). Experiments were performed in triplicate. *Bars*: SD; *P < 0.05, **P < 0.01

We further evaluated the biology function of LINC00261 in GC cells. LINC00261 was overexpressed by transfecting the pcDNA3.1-LINC00261 vector into the MGC823 cell line, which harbored the lowest expression level of LINC00261. LINC00261-overexpressing cells were selected by adding G418. In addition, LINC00261 was depleted in MGC803 cells, which exhibit high LINC00261 expression. To exclude off-target effects, we designed two different small interfering RNAs (siRNAs); both were considered appropriate for LINC00261 knockdown. The ectopic expression and knockdown of LINC00261 in the cells was confirmed by qRT-PCR (Fig. 5a). However, none of the MTT assays and cell cycle analysis detected a significant proliferative effect of LINC00261 in either the MGC803 or the BGC823 cell line (Fig. 5b, c). Subsequently, we observed the effects on cell migration and invasion. As shown in Fig. 6a, BGC823 cells, which have naturally low LINC00261 expression, after transfecting of pcDNA3.1-LINC00261 overexpression vector, exhibited a notably lower scratch-closure rate (migration inhibition) than that observed in controls infected with empty vector. Moreover, after the knockdown of LINC00261, MGC803 cells, which have naturally high LINC00261 expression, displayed a higher scratch-closure rate (migration promotion) than that in the control cells. Furthermore, cell motility was also measured using migration and invasion assays. Compared with the control cells, LINC00261-overexpressing BGC823 cells showed markedly repressed migration and invasion ability; likewise, knockdown of LINC00261 significantly stimulated migration and invasion by MGC803 cells (*P* < 0.05; Fig. 6b). These findings indicate that LINC00261 may be closely associated with invasion and migration in GC cell lines.

The article "Decreased expression of the long noncoding RNA LINC00261 indicate poor prognosis in gastric cancer and suppress gastric cancer metastasis by affecting the epithelial–mesenchymal transition" was retracted in 2018. Reasons: duplicated images; unreliable data.

**Fig. 5:** Effect of LINC00261 on gastric cancer cell proliferation and cell cycle. **a** The expression of LINC00261 in stable BGC823 cell clones infected with pcDNA3.1-LINC00261 and in MGC803 cells transfected with siRNA against LINC00261was detected by qPCR. **b** MTT assays were performed to determine the proliferation of BGC823 and MGC803 cells. **c** Cell cycle analysis determined the relative cell numbers in each cell cycle phase after propidium iodide staining of LINC00261-upregulated BGC823 cells and LINC00261-depletion MGC803 cells. *Numbers inside bars* represent percentages of cells in each phase

**Fig. 6:** Effects of LINC00261 on gastric cancer cell migration and invasion in vitro and in vivo. BGC823 cells were transfected with pcDNA3.1-LINC00261, and MGC803 cells were transfected with si-LINC00261. **a** Wound healing assays were used to investigate the migratory ability of gastric cancer cells. Experiments were performed in triplicate. *Bars*: SD; **P < 0.01. **b** Transwell assays were used to investigate changes in the migratory and invasive abilities of gastric cancer cells. Experiments were performed in triplicate. *Bars*: SD; *P < 0.05 and **P < 0.01. **c**, **d** Stable BGC823 cells transfected with pcDNA3.1-LINC00261 and an empty vector were separately injected into the tail veins of athymic mice. The lungs were harvested from the mice in each experimental group, and tumor nodules visible on lung surfaces were counted. The assay was independently conducted twice. *Bars*: SD; *P < 0.05 and **P < 0.01. **e** Visualization of the entire lung and hematoxylin and eosin (HE)-stained lung sections

The article "Decreased expression of the long noncoding RNA LINC00261 indicate poor prognosis in gastric cancer and suppress gastric cancer metastasis by affecting the epithelial–mesenchymal transition" was retracted in 2018. Reasons: duplicated images; unreliable data.

### LINC00261 suppresses GC cell metastasis in vivo

To validate the effects of LINC00261 on the metastasis of GC cells in vivo, BGC823 cells stably transfected with pcDNA3.1-LINC00261 were injected into nude mice. Metastatic nodules on the surface of the lungs were counted after 7 weeks. Ectopic overexpression of LINC00261 reduced the number of metastatic nodules compared with those in the control group (Fig. 6c, d). This difference was further confirmed following the examination of the entire lungs and through hematoxylin and eosin (HE) staining of lung sections (Fig. 6e). Our in vivo data complemented the results of the functional in vitro studies involving LINC00261.

### LINC00261 influences GC cell EMT

We conducted western blot assays to detect the expression of EMT-induced markers (E-cadherin, N-cadherin, FN1, and Vimentin) in cells overexpressing or decreasing LINC00261. Our findings showed that increased LINC00261 expression levels induced E-cadherin expression and decrease that of N-cadherin, Vimentin, and FN1, while depletion of LINC00261 inhibited E-cadherin expression and promoted N-cadherin, Vimentin, and FN1 expression (Fig. 7a). Moreover, overexpression of LINC00261 markedly increased the levels of E-cadherin, while decreasing N-cadherin and Vimentin expression in the xenograft tumors (Figs. 7b). These data support our hypothesis that LINC00261 influences the malignant phenotype by regulating EMT.

**Fig. 7:** LINC00261 overexpression suppresses GC cell invasion and metastasis by affecting the EMT. **a** Western blot analysis of E-cadherin, N-cadherin, FN1, and Vimentin expression in GC cells treated with pcDNA3.1-LINC00261 and siRNAs-LINC00261. **b** Representative E-cadherin, N-cadherin and Vimentin protein levels in xenograft tumors evaluated by immunohistochemistry. **c** Correlation analysis performed between E-cadherin, N-cadherin, and Vimentin expression levels and the different xenograft tumor groups

## Discussion

Many lncRNAs have been implicated in various types of cancers. Reportedly, the lncRNAs of the class MALAT-1 have been found to promote cell motility in lung adenocarcinoma cells [17]. PCGEM1 overexpression and PRNCR1 have been found to be involved in the development of prostate cancer [18, 19]. Recent findings have also suggested that many lncRNAs have important roles in GC. MALAT1 and HOTAIR were recently reported to drive GC development and promote peritoneal metastasis. Xu et al. revealed that the lncRNA FENDRR inhibits invasive and metastatic behavior in GC cells [10]. TINCR was reported to promote GC proliferation by accelerating KLF2 mRNA degradation [11]. Therefore, the identification of GC-associated lncRNAs may provide a missing piece of the well-known oncogenic and tumor suppressor network puzzle.

The article "Decreased expression of the long noncoding RNA LINC00261 indicate poor prognosis in gastric cancer and suppress gastric cancer metastasis by affecting the epithelial–mesenchymal transition" was retracted in 2018. Reasons: duplicated images; unreliable data.

Previous profiling study identified that LINC00261 was downregulated in GC tissues compared to normal tissue samples [14]. However, its function in carcinogenesis and tumor progression is unclear. In this study, we confirmed that LINC00261 levels were decreased in GC cells and tissues compared with the normal gastric epithelial cells and adjacent normal tissues. LINC00261 can serve as a biomarker to distinguish cancer tissue with non-tumor tissue in GC. Moreover, low LINC00261 expression was significantly correlated with aggressive tumor characteristics (greater invasion depth, higher tumor stage, and lymphatic metastasis) and poor prognosis. When the patients were subdivided into four groups according to tumor stage, we found that LINC00261 expression could distinguish patients with different outcomes in stages III and IV. However, we did not observe a significant correlation between LINC00261 expression and clinical outcomes in the early clinical stages of GC, probably due to better outcome in the early stage of GC after treatment of operation. Univariate and multivariate analyses indicated that DFS were significantly better among patients with high LINC00261 expression than in patients with low LINC00261 expression in the same stage. Multivariate analysis demonstrated that LINC00261 expression was an independent prognostic factor for GC patients. This suggests that LINC00261 might be a promising prognostic and diagnostic biomarker in GC patients.

As low LINC00261 expression was associated with an aggressive tumor phenotype in GC, we speculated that LINC00261 could play a significant role in tumor biology. Initially, we chose representative cell lines of GC and investigated their LINC00261 expression in comparison to a non-tumoral gastric cell line. We observed that all of the five tumor cell lines exhibited low LINC00261 expression, which corroborated our previous findings. We next determined whether LINC00261 expression influenced tumor-like characteristics, such as proliferation and metastasis. Ectopic expression of LINC00261 inhibited cell migration and invasion, whereas knockdown of endogenous LINC00261 expression significantly enhanced these capacities. Moreover, increased LINC00261 expression significantly reduced the number of metastatic nodules on the lungs in vivo. However, no significant effect on cellular proliferation was observed after ectopic expression or knockdown of LINC00261. This is in line with our clinical findings that LINC00261 was significantly correlated with invasion depth, tumor stage, and lymphatic metastasis, but not tumor size. These results revealed that LINC00261 might impact the prognosis of GC by affecting cell migration and invasion.

The article "Decreased expression of the long noncoding RNA LINC00261 indicate poor prognosis in gastric cancer and suppress gastric cancer metastasis by affecting the epithelial–mesenchymal transition" was retracted in 2018. Reasons: duplicated images; unreliable data.

To explore the molecular mechanism through which LINC00261 contributes to invasion and metastasis in GC, we investigated potential target proteins involved in cell motility and matrix invasion. The EMT plays crucial roles during cancer initiation and progression, especially in cancer metastasis [20–22]. Previous data has been revealed that lncRNAs regulate tumor cell metastasis by affecting the EMT process [23, 24]. Hallmarks of EMT are the loss of E-cadherin expression and the aberrant expression of N-cadherin and Vimentin. Therefore, we determined the levels of these EMT-induced markers following overexpression or inhibition of LINC00261. Our results indicated that LINC00261 mediated inhibitory effects on GC cell metastasis suppression, possibly by affecting the EMT. As a central differentiation process, EMT allows for the remodeling of tissues during the early stages of embryogenesis and is implicated in the promotion of tumor cell invasion and metastasis. Therefore, as regulators of EMT, lncRNAs could be suitable candidates for intervention in the treatment of cancer. In recent years, molecularly targeted therapeutics for key molecular drivers of cancer progression has been developed [25]. LINC00261, as an important regulator of EMT, promise to serve as a drug target. Drugs which could regulate the expression of LINC00261 have clinical application prospects, so clinical test or assay could be developed to test these.

## Conclusions

In summary, our study showed that LINC00261 is dramatically downregulated in GC tissues and cell lines and that the low expression of LINC00261 is significantly associated with invasion depth, tumor stage, lymphatic metastasis, and patients’ survival time. Moreover, upregulation of LINC00261 has the effect of suppressing GC cell migration and invasion in vitro and in vivo by targeting EMT markers. Further insights into the functional and clinical implications of LINC00261 and its targets may help with the treatment of GC.

## Methods

### Computational analysis

Human microarray datasets were downloaded from NCBI’s Gene Expression Omnibus (GEO, http://www.ncbi.nlm.nih.gov/geo/) and are accessible through GEO series accession number GSE13911. GEO database and background were adjusted using Robust Multichip Average. GATExplorer was used to process microarrays on a local computer for gene expressions of lncRNAs [26]. This GATExplorer provides a series of R packages, designed to be used with BioConductor tools, which allow applying in a simple way the probe mapping data included in GATExplorer. A type of files called ncRNA Mapper was also obtained from GATExplorer, which includes the probes that do not map to any coding region but that were mapped to a database for ncRNA of human and mouse derived from RNAdb [27]. A customized R script was used to perform a microarray expression calculation according to the re-mapping data (file ncrnamapperhgu133plus2cdf_3.0) obtained from public database NCBI.

The article "Decreased expression of the long noncoding RNA LINC00261 indicate poor prognosis in gastric cancer and suppress gastric cancer metastasis by affecting the epithelial–mesenchymal transition" was retracted in 2018. Reasons: duplicated images; unreliable data.

The online software including ORF Finder (http://www.ncbi.nlm.nih.gov/gorf/gorf.html), PhyloCSF (https://github.com/mlin/PhyloCSF/wiki), and Coding Potential Calculator (CPC; http://cpc.cbi.pku.edu.cn/) were used to assessment of lncRNA protein-coding potential.

To gain further insight into the biologic pathways involved in GC pathogenesis through LINC00261 pathway, a Gene Set Enrichment Analysis (GSEA) was performed. The gene sets showing FDR of 0.25, a well-established cutoff for the identification of biologically relevant gene, were considered enriched between classes under comparison.

### 5′ and 3′ rapid amplification of cDNA ends (RACE) analysis

We used the 5′ and 3′ RACE analyses to determine the transcriptional initiation and termination site of GCASPC using a SMARTer RACE cDNA Amplification kit (Clontech, Palo Alto, CA, USA), according to the manufacturer’s instructions. PCR of the internal region was performed when starting points of 5′ and 3′ RACE had an unamplified gap. RACE PCR products were separated on a 1.5 % agarose gel. Gel products were extracted with the Gel and PCR Clean-Up System (Promega, A9282), cloned into the pGEM-T Vector Systems I (Promega, A3600) and sequenced bidirectionally using the M13 forward and reverse primers by Sanger sequencing at Invitrogen. At least five colonies were sequenced for every RACE PCR product that was gel purified.

### Cell lines

The human gastric adenocarcinoma cell lines MGC803, BGC823, MKN28, MKN45, and SGC7901 and the normal gastric epithelial cell line (GES-1) were obtained from the Chinese Academy of Sciences Committee on Type Culture Collection cell bank (Shanghai, China). MGC803, BGC823, and MKN28 cells were cultured in Roswell Park Memorial Institute (RPMI) 1640 medium; MKN45, GES-1, and SGC7901 cells were cultured in a Dulbecco-modified Eagle medium (DMEM; GIBCO-BRL) supplemented with 10 % fetal bovine serum (FBS), 100 U/ml penicillin, and 100 mg/ml streptomycin (Invitrogen, Carlsbad, CA, USA) at 37 °C in 5 % CO_2_.

The article "Decreased expression of the long noncoding RNA LINC00261 indicate poor prognosis in gastric cancer and suppress gastric cancer metastasis by affecting the epithelial–mesenchymal transition" was retracted in 2018. Reasons: duplicated images; unreliable data.

### Tissue samples and clinical data collection

In this study, we analyzed 138 patients who underwent resection of primary GC at the 1st Affiliated Hospital of Wenzhou Medical University, the affiliated People’s Hospital of Jiangsu University, and the First People’s Hospital of Yangzhou. All the patients were treated by 5-fluorouracil (5-FU)-based chemotherapy after gastrectomy: oxaliplatin, leucovorin, and 5-FU (modified FOLFOX) for 6 cycles. The study was approved by the Ethics Committee on Human Research of the 1st Affiliated Hospital of Wenzhou Medical University, the affiliated People’s Hospital of Jiangsu University, and the First People’s Hospital of Yangzhou, and written informed consent was obtained from all the patients. The clinicopathological characteristics of the GC patients are summarized in Table 1. All patients with GC have been followed up at intervals of 1–2 months until April 2016, and the median follow-up period was 36 months (range, 20–48 months). Follow-up studies included physical examination, laboratory analysis, and computed tomography if necessary. DFS was defined as the interval between the dates of surgery and recurrence; if recurrence was not diagnosed, patients were censored on the date of death or the last follow-up.

### RNA preparation and quantitative real-time PCR

Total RNAs were extracted from tumorous and adjacent normal tissues or cultured cells using Trizol reagent (Invitrogen) following the manufacturer’s protocol. RT and qPCR kits (Takara, Dalian, China) were used to evaluate the expression of LINC00261 in tissue samples and cultured cells. The primers used in this study are shown in Additional file 4: Table S1. Real-time PCR was performed in triplicate, and the relative expression of LINC00261 was calculated using the comparative cycle threshold (2^−ΔΔCT^) method with glyceraldehyde-3-phosphate dehydrogenase (GAPDH) as the endogenous control to normalize the data.

### Vector construction and transfection and siRNA transfection

To overexpress LINC00261, the coding sequence of LINC00261 was amplified and subcloned into the pcDNA3.1 (+) vector (Invitrogen) according to the manufacturer’s instructions. BGC823 cells were then transfected with a negative control vector or the LINC00261-expressing plasmid using Lipofectamine 2000 (Invitrogen). To generate LINC00261 knockdown MGC803 cells, the target sequence for LINC00261 siRNA or scrambled siRNA that did not correspond to any human sequence was synthesized (Invitrogen). The siRNA sequences are shown in Additional file 4: Table S1.

### Cell proliferation assays

Cell viability was monitored using a Cell Proliferation Reagent Kit I (MTT; Roche Applied Science). MGC803 cells transfected with si-LINC00261 (3000 cells/well) and BGC823 cells transfected with Pcdna3.1-LINC00261 were grown in 96-well plates. Cell viability was assessed every 24 h following the manufacturer’s protocol. All experiments were performed in quadruplicate. For colony formation assays, Pcdna3.1-LINC00261-transfected BGC823 cells (*n* = 500) were placed in 6-well plates and maintained in media containing 10 % FBS. The medium was replaced every 4 days; after 14 days, the cells were fixed with methanol and stained with 0.1 % crystal violet (Sigma-Aldrich). Visible colonies were then counted. For each treatment group, wells were assessed in triplicate, and experiments were independently repeated three times.

The article "Decreased expression of the long noncoding RNA LINC00261 indicate poor prognosis in gastric cancer and suppress gastric cancer metastasis by affecting the epithelial–mesenchymal transition" was retracted in 2018. Reasons: duplicated images; unreliable data.

### Wound healing assay

For the wound healing assay, 3 × 10^5^ cells were seeded in 6-well plates, cultured overnight, and transfected with pCDNA3.1-LINC00261, si-LINC00261, or a control. Once cultures reached 85 % confluence, the cell layer was scratched with a sterile plastic tip and washed with culture medium. The cells were then cultured for 48 h with medium containing 1 % FBS. At different time points, images of the plates were acquired using a microscope. The distance between the two edges of the scratch was measured using the Digimizer software system. The assay was independently repeated three times.

### Cell migration and invasion assays

For the migration assays, at 48 h post-transfection, 5 × 10^4^ cells in serum-free media were placed into the upper chamber of an insert (8-μm pore size; Millipore). For the invasion assays, 1 × 10^5^ cells in a serum-free medium were placed into the upper chamber of an insert coated with Matrigel (Sigma-Aldrich). The medium containing 10 % FBS was added to the lower chamber. After incubation for 24 h, the cells remaining on the upper membrane were removed with cotton wool. Cells that had migrated or invaded through the membrane were stained with methanol and 0.1 % crystal violet, imaged, and counted using an IX71 inverted microscope (Olympus, Tokyo, Japan). Experiments were independently repeated three times.

### Western blot assay and antibodies

Cells were lysed using radioimmunoprecipitation assay protein extraction reagent (Beyotime, Beijing, China) supplemented with a protease inhibitor cocktail (Roche, CA, USA) and phenylmethylsulfonyl fluoride (Roche). The concentration of proteins was determined using a Bio-Rad protein assay kit. Protein extracts (50 μg) were separated by 10 % sodium dodecyl sulfate–polyacrylamide gel electrophoresis (SDS-PAGE), transferred to nitrocellulose membranes (Sigma), and incubated with specific antibodies. Electrochemiluminescent chromogenic substrate was used to visualize the bands, and the intensity of the bands was quantified by densitometry (Quantity One software; Bio-Rad), with GAPDH used as a control. Antibodies (1:1000 dilutions) against E-cadherin, N-cadherin, FN1, and Vimentin were purchased from BD.

The article "Decreased expression of the long noncoding RNA LINC00261 indicate poor prognosis in gastric cancer and suppress gastric cancer metastasis by affecting the epithelial–mesenchymal transition" was retracted in 2018. Reasons: duplicated images; unreliable data.

### Metastasis assay in athymic mouse model

Male athymic mice (4 weeks old) were purchased from the Animal Center of the Chinese Academy of Science (Shanghai, China) and maintained in laminar flow cabinets under specific pathogen-free conditions. BGC823 cells transfected with pCDNA3.1-LINC00261 or the empty vector were harvested from 6-well plates, washed with phosphate-buffered saline (PBS), and resuspended at a density of 2 × 10^7^ cells/ml. The cell suspension (0.1 ml) was injected into the tail veins of 10 mice, which were sacrificed 7 weeks after the injection. Metastasis focuses appeared mostly in the lung upon tail vein injection of athymic mouse [10]. So the lungs were removed and photographed, and visible tumors on the lung surface were counted. This study was carried out in strict accordance with the Guide for the Care and Use of Laboratory Animals of the National Institutes of Health. Our protocol was approved by the Committee on the Ethics of Animal Experiments of Wenzhou Medical University. All surgery was performed under sodium pentobarbital anesthesia, and all efforts were made to minimize suffering [28]. The metastasis assays in athymic mice were independently performed for two replicates.

### Immunohistochemical analysis

The immunohistochemical analysis of E-cadherin, N-cadherin, and Vimentin was performed according to a previously described method [29]. Immunohistochemical score was semiquantitatively evaluated on the basis of staining intensity and distribution using the immunoreactive score: intensity score× proportion score. The staining intensity was scored as follows: 0, negative; 1, weak; 2, moderate; or 3, strong. The proportion score was defined as follows: 0, negative; 1, 10 % or less; 2, 11 to 50 %; 3, 51 to 80 %; or 4, 80 % or more positive cells. The total score ranged from 0 to 12. The immunoreactivity was divided into three levels on the basis of the final score: negative expression was defined as a total score of 0; low expression, as a total score of 1 to 4; and high expression, as a total score higher than 4. Immunoreactivity was assessed independently by two investigators who were blinded to the other immunohistochemical results.

### Statistical analysis

All statistical analyses were performed using SPSS 20.0 software (IBM, SPSS, Chicago, IL, USA). The significance of the differences between groups was estimated by Student’s *t* test, *χ*^2^ test, or Wilcoxon test, as appropriate. DFS rates were calculated by the Kaplan–Meier method with the log-rank test applied for comparison. Survival data were evaluated using univariate and multivariate Cox proportional hazards models. Variables with a value of *P* < 0.05 in univariate analysis were used in subsequent multivariate analysis on the basis of Cox regression analyses. Pearson correlation analyses were performed to investigate the correlation among LINC00261 with E-cadherin, N-cadherin, and FN1 expressions. Two-sided *P* values were calculated, and a probability level of 0.05 was chosen for statistical significance.

The article "Decreased expression of the long noncoding RNA LINC00261 indicate poor prognosis in gastric cancer and suppress gastric cancer metastasis by affecting the epithelial–mesenchymal transition" was retracted in 2018. Reasons: duplicated images; unreliable data.

## Abbreviations

DFS, disease-free survival; EMT, epithelial–mesenchymal transition; FN1, Fibronectin1; GC, gastric cancer; HR, hazard ratio; lncRNA, long noncoding RNA; MMPs, matrix metalloproteinases; PCR, polymerase chain reaction

## Additional files

Additional file 1: Table S2 Clinical data of all patients involved in the study. (XLS 40 kb) Additional file 2: Table S3 cDNA sequence of two isoforms of LINC00261 identified by the RACE assay. (DOC 36 kb) Additional file 3: Table S4 Top-scoring genes which is enriched in the focal adhesion pathway according to LINC00261 expression. (XLS 10 kb) Additional file 4: Table S1 Primers used for qRT-PCR and siRNA oligonucleotides. (XLS 16 kb)
